# Functional Consequences of a Novel Variant of *PCSK1*

**DOI:** 10.1371/journal.pone.0055065

**Published:** 2013-01-28

**Authors:** Lindsay A. Pickett, Michael Yourshaw, Valeria Albornoz, Zijun Chen, R. Sergio Solorzano-Vargas, Stanley F. Nelson, Martín G. Martín, Iris Lindberg

**Affiliations:** 1 Department of Human Genetics, David Geffen School of Medicine, University of California Los Angeles, Los Angeles, California, United States of America; 2 Division of Gastroenterology and Nutrition, Department of Pediatrics, Mattel Children's Hospital and David Geffen School of Medicine, University of California Los Angeles, Los Angeles, California, United States of America; 3 Department of Anatomy and Neurobiology, University of Maryland-Baltimore, Baltimore, Maryland, United States of America; 4 Department of Pathology and Laboratory Medicine, David Geffen School of Medicine, University of California Los Angeles, Los Angeles California, United States of America; National Cancer Institute, National Institutes of Health, United States of America

## Abstract

**Background:**

Common single nucleotide polymorphisms (SNPs) in proprotein convertase subtilisin/kexin type 1 with modest effects on PC1/3 *in vitro* have been associated with obesity in five genome-wide association studies and with diabetes in one genome-wide association study. We here present a novel SNP and compare its biosynthesis, secretion and catalytic activity to wild-type enzyme and to SNPs that have been linked to obesity.

**Methodology/Principal Findings:**

A novel PC1/3 variant introducing an Arg to Gln amino acid substitution at residue 80 (within the secondary cleavage site of the prodomain) (rs1799904) was studied. This novel variant was selected for analysis from the 1000 Genomes sequencing project based on its predicted deleterious effect on enzyme function and its comparatively more frequent allele frequency. The actual existence of the R80Q (rs1799904) variant was verified by Sanger sequencing. The effects of this novel variant on the biosynthesis, secretion, and catalytic activity were determined; the previously-described obesity risk SNPs N221D (rs6232), Q665E/S690T (rs6234/rs6235), and the Q665E and S690T SNPs (analyzed separately) were included for comparative purposes. The novel R80Q (rs1799904) variant described in this study resulted in significantly detrimental effects on both the maturation and *in vitro* catalytic activity of PC1/3.

**Conclusion/Significance:**

Our findings that this novel R80Q (rs1799904) variant both exhibits adverse effects on PC1/3 activity and is prevalent in the population suggests that further biochemical and genetic analysis to assess its contribution to the risk of metabolic disease within the general population is warranted.

## Introduction

Prohormone convertase 1/3 is a calcium-dependent serine endoprotease essential for the conversion of a variety of prohormones and neuropeptide precursors to their bioactive forms. Human prohormone convertase 1/3 (PC1/3) is encoded by the gene *PCSK1*, which is located on chromosome 5 and is comprised of 14 exons [1]. PC1/3 is expressed in a subset of endocrine and neuroendocrine tissues, cells equipped with a regulated secretory pathway. During transit through the secretory pathway, PC1/3 is first synthesized in the endoplasmic reticulum (ER) as an inactive 94 kDa zymogen composed of an N-terminal signal peptide, a prodomain which serves as an intramolecular chaperone and inhibitor; a catalytic domain which accomplishes substrate hydrolysis; a P (homo B) domain which contributes to enzymatic properties; and a carboxyl-terminal (CT) domain which, when removed by partial or complete *in trans* proteolytic processing, results in a much more active, but also less stable, enzymatic form (reviewed in [2] (**Figure 1**). PC1/3 is abundantly expressed in the arcuate and paraventricular nuclei of the hypothalamus [3], [4], tissues that are known to mediate satiety and hunger signals [5]. Substrates of PC1/3, such as proinsulin, proglucagon, proghrelin, agouti-related protein, pro-neuropeptide Y, provasopressin and proopiomelanocortin are responsible for the regulation of absorption, metabolism and acquisition (appetite) of nutrients [6], [7], [8], [9], [10], [11], [12], [13], [14].

**Figure 1:** Domain structure and SNP locations within preproPC1/3. The upward arrows indicate the cleavage sites required for PC1/3 maturation. The downward arrows indicate locations of previously described (black) and novel (purple) SNP. The dashed line between the pro and catalytic domains represents a primary cleavage site (occurring in the ER) that is required for activation. The dashed line in the middle of the prodomain indicates the secondary cleavage site (likely cleaved in the trans-Golgi network). The P or Homo B domain following the catalytic domain is important for the stabilization of the catalytic domain, as well as determining various enzymatic properties. The C-terminal domain plays a role in efficient routing of PC1/3 to the secretory granules, and contributes to substrate specificity as well as to specific activity and stability.

Deficiencies in PC1/3 frequently lead to imbalances in prohormone processing that result in an array of metabolic phenotypes, previously investigated both in mouse models and in humans. Three human subjects have been described with an autosomal recessive disorder (MIM:600955) associated with severe mutations of PC1/3 resulting in early-onset obesity, hyperphagia, hypoadrenalism, reactive hypoglycemia, malabsorptive diarrhea, and hypogonadism [15], [16], [17]. Interestingly, the PC1/3 null mouse model, unlike the PC1/3-deficient human, is not obese. Although of normal weight at birth, PC1/3 null mice have a high post-natal mortality rate, and those that do survive have a significant reduction in body mass as compared to wild-type animals by the age of 6 weeks. The stunted growth of PC1/3 null mice is believed to be due at least in part to reduced processing of growth hormone releasing hormone (GHRH) and thus reduced circulating levels of growth hormone (GH) [8]. In addition to a reduction in GHRH, the levels of several key neuroendocrine peptides such as ACTH, insulin and glucagon-like peptides-1 and -2 are reduced in these animals due to lack of precursor processing by PC1/3 [8].

While the PC1/3 null mouse is not obese, a mouse model of obesity has been generated via introduction of a missense mutation in *PCSK1* at amino acid position 222, near the calcium-binding pocket in the catalytic domain. This hypomorph mutation resulted in obesity, hyperphagia and increased metabolic efficiency due to decreased autocatalytic maturation of the enzyme to smaller molecular weight forms [18]. Three common SNPs in *PCSK1* have been identified and associated with obesity. All three SNPs (included in this study for comparison) exhibit moderate effects on catalytic activity *in vitro* and on natural substrate processing in rat pituitary tumor cells [19], [20]. Two of the three non-deleterious SNPs (S690T [rs6235] and Q665E [rs6234]) have been associated with diabetes-related traits [20], [21], [22].

In the work presented below, the novel variant NP_000430.3:p.Arg80Gln (R80Q; rs1799904), identified and functionally evaluated for the first time here, was compared with previously described SNPs associated with obesity and/or diabetes (N221D [rs6232], Q665E/S690T [rs6234/rs6235], Q665E [rs6234], and S690T [rs6235]) for potentially deleterious effects on the biosynthesis, secretion and catalytic activity of PC1/3. Our data suggest that this novel R80Q variant (rs1799904) deserves further analysis to assess its genetic association with metabolic diseases such as obesity and diabetes.

## Materials and Methods

### Databases used and protein structure/function analysis methods

Alleles that varied from the human reference genome build GRCh37 [23] were obtained from the dbSNP [24], 1000 Genomes [25], NHLBI [26], and NIEHS [27] datasets and were merged into a custom SQL database. dbSNP data were compiled from various sources, with allele frequencies available only for a subset of variants. The 1000 Genomes dataset was based on both low coverage whole genome and higher coverage exome sequencing of 1092 individuals. The NHLBI and NIEHS data were obtained from exome sequencing of 6500 and 95 individuals respectively. Population allele frequencies were calculated using the combined datasets wherever allele counts were present. Variations in *PCSK1* (chr5:95726119-95769847) were identified and analyzed with the Ensembl Variant Effect Predictor version 2.6 [28] and Ensembl database homo_sapiens_variation_68_37 [29] to determine the effect of the variant on the transcript. Non-synonymous codon substitutions were analyzed using the SIFT [23], [30], [31], [32], [33], PolyPhen [34], [35], [36], and Condel [37] models to estimate the variant's probable impact on protein structure and function.

### Sanger sequencing of genomic DNA

Genomic DNA from individuals homozygous for two SNPs of interest was isolated from EBV-infected B cells by the Coriell Institute and sent to us for sequencing. The HG00596 DNA sample containing rs1799904 (p.R80Q; (g.5:95764963C>T; c.239G>A) was obtained from a southern Han Chinese female, while the N586Tfsx4-containing (g.5:95730696TC>T; c.1755delG) DNA sample, HG00350, was obtained from a Finnish female. The primers used for sequencing bidirectionally were:

Exon 2 (510 bp):

(F) CTCAACCAATTCAACCCAATC;

(R) CCCGTGACACAAGTTTACCTATG; and

Exon 13 (545 bp):

(F) CAGCTTTCCAAGAACACATCC;

(R) CCATGTTTGACTTATTTCCTGC

### Expression vector construction/mutagenesis

Flag-tagged human PC1/3, a kind gift of J. W. Creemers [20] was modified by site-directed mutagenesis using the Stratagene QuikChange method [38] to introduce the mutations shown in **Figure 1**. All mutations were verified by sequencing of the entire PC1/3 cDNA insert.

### Transient transfection of PC1/3 variants

To assess the biosynthesis and secretion profiles of PC1/3 variants in a cell line that does not express endogenous PC1/3, Ad-293 (Stratagene) HEK cells, plated at a density of 2×10^5^ cells per well in 24-well plates, were transfected with plasmids encoding either wild-type or variant PC1/3s in triplicate wells. Cells were transfected with 200 ng of plasmid DNA per well using Lipofectamine (Invitrogen, Carlsbad, CA). To assess effects in a regulated neuroendocrine cell line (also lacking expression of endogenous PC1/3), Neuro-2A cells (ATCC, cat. No. CCL-131) were transfected in triplicate with the same protocol using Lipofectamine 2000 (Invitrogen, Carlsbad, CA). For both cell lines, five hours post-transfection, 1 ml of growth medium was added to each well and incubation continued for an additional 24 h. Cells were then washed with PBS and 0.3 ml of Opti-MEM (Invitrogen, Carlsbad, CA) containing 100 ug/ml bovine aprotinin (Desert Biologicals) was added to each well. Cells were incubated for an additional 18–24 h before conditioned medium and cells were harvested. Conditioned medium was analyzed first by enzyme assay; both cells and medium samples (for HEK cells) and medium samples (for Neuro- 2A cells) were then subjected to SDS-PAGE followed by Western blotting using primary antiserum against the amino terminus of mature mouse PC1/3 [39]. Mouse monoclonal anti-ß-actin antiserum (Sigma-Aldrich, St. Louis, MO) was used to assess cellular actin levels as a loading control. Western blots were then probed with horseradish peroxidase-coupled secondary antiserum. Visualization of immunoreactive protein was accomplished using the SuperSignal West Femto Maximum Sensitivity Substrate kit (Thermo Scientific, Rockford, IL).

### Enzyme assay

Enzymatic activity of secreted recombinant PC1/3 proteins present in conditioned medium obtained from transiently transfected HEK293 cells was measured in triplicate 50 ul reactions in a 96-well polypropylene plate containing 25 ul of conditioned medium and final concentrations of 200 uM substrate (pyr-ERTKR-amc [7-amino-4-methlcoumarin]), 100 mM sodium acetate, pH 5.5, 2 mM CaCl_2_, 0.1% Brij 35, and a protease inhibitor cocktail (final concentrations: 1 uM pepstatin, 0.28 mM TPCK, 10 uM E-64, and 0.14 mM TLCK). Reaction mixtures were incubated at 37°C and fluorescence measurements (380 nm excitation, 460 emission) were taken under kinetic conditions every 20 seconds for 1 h in a SpectraMax M2 Microplate Reader. Maximum rates were obtained from the linear portion of the kinetic measurement curves. Specific activities of PC1/3 proteins in the conditioned medium were determined by dividing maximum rates by band intensities of total secreted immunoreactive protein, each determined in triplicate, and quantified with an Alphaimager 3300 (Alpha Innotech Corporation, San Leandro, CA) imaging system.

## Results

### Analysis of public databases; structure-function analysis

A total of 1020 allelic variants (data not shown) within the *PCSK1* gene were found in the public databases, of which 54 were potentially consequential splice site or missense variants (**Table 1**). Thirty-seven non-synonymous substitutions were predicted to be possibly or probably deleterious by at least one model (SIFT, PolyPhen, or Condel, where Condel represents a consensus modeling program). Two of the three previously described variants are common, with MAFs of 23.7% for S690T (rs6235) and 25.0% for Q665E (rs6234), whereas the N221D SNP (rs6232) is less common (MAF = 3.3%). None of these three variants were predicted to be deleterious using SIFT, PolyPhen, or Condel. In contrast, the novel variants that were predicted as “possibly” or “probably” deleterious were unique to one sample or were observed with very low frequency (minor allele frequencies (MAFs) of 0.008%–0.87%. In addition we considered a frameshift variant N586TfX4 (g.5:95730696), which exhibited an unusually large MAF of 6.1% in a previous release of the 1000 Genomes data. We selected the most common novel variant R80Q (rs1799904; MAF = 0.87%), and N586TfsX4 for genomic sequencing and potential functional studies, comparing them with already described common variants of PC1/3.

**Table 1:** Potentially consequential variant alleles in *PCSK1*.

Pos	ID	REF	ALT	Rank	cDNA	Protein	Effect	MAF	Samples	Het	Hom
5:95768682	rs201377789	A	G	12	65T>C	Leu22Pro		0.00033	7690	5	0
5:95764976		G	A	12	226C>T	Pro76Ser		0.00008	6501	1	0
5:95764968	rs148354360	C	A	12	234G>T	Arg78Ser	SpC	0.00015	6501	2	0
**5:95764963**	**rs1799904**	**C**	**T**	**12**	**239G>A**	**Arg80Gln**	**p**	**0.00870**	**1092**	**17**	**1**
5:95761576	rs200893367	T	G	12	344A>C	Asp115Ala	S	0.00046	1092	1	0
5:95761546		A	T	12	374T>A	Met125Lys		0.00008	6503	1	0
5:95761545	rs146545244	C	T	12	375G>A	Met125Ile		0.00038	6503	5	0
5:95759156		G	A	12	404C>T	Thr135Ile	PC	0.00008	6503	1	0
5:95759151		T	G	12	409A>C	Met137Leu		0.00008	6503	1	0
5:95759098	rs145659863	T	G	12	462A>C	Lys154Asn	S	0.00008	6503	1	0
5:95759093		A	G	12	467T>C	Ile156Thr	SpC	0.00008	6503	1	0
5:95759090	rs200462856	G	A	12	470C>T	Thr157Met	SPC	0.00015	6503	2	0
5:95759036	rs140520429	G	A	12	524C>T	Thr175Met	SPC	0.00026	7595	4	0
5:95759019	rs145592525	A	G	12	541T>C	Tyr181His	SPC	0.00038	6503	5	0
5:95757611		G	A	12	593C>T	Pro198Leu	SPC	0.00008	6503	1	0
5:95751796	rs202203086	G	A	12	650C>T	Ala217Val	SPC	0.00013	7595	2	0
*5:95751785*	*rs6232*	*T*	*C*	*12*	*661A>G*	*Asn221Asp*		*0.03289*	*8254*	*523*	*10*
5:95751745	rs145127903	T	A	12	701A>T	Lys234Ile	SPC	0.00008	6503	1	0
5:95751742	rs183045011	A	G	12	704T>C	Val235Ala	SPC	0.00046	1092	1	0
5:95748134		T	C	12	770A>G	Asn257Ser	S	0.00008	6503	1	0
5:95748123		C	T	12	781G>A	Val261Met	SPC	0.00008	6503	1	0
5:95748122	rs139602265	A	G	12	782T>C	Val261Ala	SPC	0.00008	6503	1	0
5:95748068	rs142673134	C	G	12	836G>C	Gly279Ala	SPC	0.00008	6503	1	0
5:95748035	rs193214131	T	C	12	869A>G	Tyr290Cys	PC	0.00026	7595	4	0
5:95746664		G	C	12	909C>G	Phe303Leu	SPC	0.00008	6503	1	0
5:95746663	rs148617898	C	T	12	910G>A	Val304Ile	pC	0.00038	6503	5	0
5:95746638	rs138879299	C	T	12	935G>A	Arg312His	S	0.00008	6503	1	0
5:95746543	rs189927028	C	T	12	1030G>A	Ala344Thr	P	0.00046	1092	1	0
5:95744026		G	A	12	1097C>T	Thr366Met	S	0.00008	6503	1	0
5:95735742	rs140481124	G	C	12	1345C>G	Leu449Val	SPC	0.00008	6503	1	0
5:95735724		G	T	12	1363C>A	Pro455Thr	SpC	0.00008	6503	1	0
5:95735703	rs151257336	G	T	12	1384C>A	Pro462Thr	SpC	0.00008	6503	1	0
5:95735700	rs143174906	C	T	12	1387G>A	Glu463Lys		0.00059	7595	9	0
5:95734621	rs149124467	C	T	12	1550G>A	Arg517Gln	pC	0.00015	6503	2	0
5:95734610		G	A	12	1561C>T	Leu521Phe	SpC	0.00008	6503	1	0
5:95734581		A	G	3	1588+2T>C		-	0.00015	6503	2	0
5:95730719	rs145196120	A	G	12	1733T>C	Ile578Thr		0.00008	6503	1	0
5:95730638		C	T	12	1814G>A	Arg605His	SPC	0.00008	6503	1	0
5:95730629		G	A	12	1823C>T	Thr608Met	SpC	0.00015	6503	2	0
5:95730597	rs144324144	C	G	12	1855G>C	Gly619Arg	P	0.00008	6503	1	0
5:95730576		G	T	12	1876C>A	Pro626Thr		0.00008	6503	1	0
5:95729049	rs139453594	T	C	12	1918A>G	Thr640Ala		0.00145	7595	22	0
5:95729048	rs193015519	G	A	12	1919C>T	Thr640Ile		0.00013	7595	2	0
5:95729039	rs142453906	G	C	12	1928C>G	Ser643Cys		0.00008	6502	1	0
5:95729007	rs200614230	G	A	12	1960C>T	Arg654Trp	S	0.00046	1092	1	0
5:95728982	rs148807505	G	T	12	1985C>A	Ala662Asp	S	0.00008	6503	1	0
*5:95728974*	*rs6234*	*G*	*C*	*12*	*1993C>G*	*Gln665Glu*		*0.24962*	*7900*	*2988*	*478*
*5:95728898*	*rs6235*	*C*	*G*	*12*	*2069G>C*	*Ser690Thr*		*0.23747*	*7900*	*2852*	*450*
5:95728877	rs138433207	T	G	12	2090A>C	Tyr697Ser		0.00008	6503	1	0
5:95728863	rs140899352	C	T	12	2104G>A	Glu702Lys		0.00039	7595	6	0
5:95728862	rs188666266	T	G	12	2105A>C	Glu702Ala	S	0.00046	1092	1	0
5:95728749		G	A	12	2218C>T	Arg740Trp	SPC	0.00008	6503	1	0
5:95728748	rs140941383	C	T	12	2219G>A	Arg740Gln	SPC	0.00008	6503	1	0
5:95728710	rs147016634	T	G	12	2257A>C	Asn753His	SC	0.00046	7595	7	0

The R80Q (rs1799904) variant that differed from the human reference genome and was predicted to have a potentially consequential effect on the transcript was selected from the dbSNP 137, 1000 Genomes, NHLBI, and NIEHS public datasets. *Pos*: genomic position in GRCh37; *ID*: dbSNP 137 rs ID; *REF*: reference allele; *ALT*: alternate allele (variant); *Rank*: 3 splice_donor_variant, 12 missense_variant; *cDNA*: position and consequence of variant in cDNA of canonical NM_000439.4 transcript; *Protein*: position and consequence of variant in NP_000430.3 protein; *Effect*: computational prediction of effect on protein structure or function (“S” predicted deleterious by SIFT, “P” or “p” predicted probably or possibly damaging by PolyPhen, “C”, predicted deleterious by Condel from a consensus of SIFT and PolyPhen, “-” no prediction); *MAF*: minor allele frequency across all populations; *Samples*: total number of individuals genotyped; *Het*: number of individuals heterozygous for the variant allele; *Hom*: number of individuals homozygous for the variant allele. Known, common variants are listed in italics, and the rare novel variant is shown in bold.

### SNP validation by sequencing

Genomic DNA from two individuals homozygous for the most common variants was obtained from the Coriell Institute and subjected to Sanger sequencing. The DNA sample containing rs1799904 (R80Q (g.5:95764963C>T; c.239G>A) was found to be homozygous for the R80Q mutation in exon 2 (**Figure 2**), while the N586Tfsx4-containing SNP (g.5:95730696TC>T; c.1755delG) was determined to be a false positive (*i.e.* no frameshift mutation was found in in exon 13) (data not shown).

**Figure 2:** Direct Sanger sequencing of genomic DNA from a subject bearing the Arg80Gln variant.

### Secretion and biosynthesis of PC1/3 variants

In order to assess whether the novel variant R80Q (rs1799904) affected the biosynthesis or secretion of PC1/3, expression vectors encoding wild-type and variant *PCSK1*s were transiently transfected into HEK and/or Neuro-2a cells (both lines lack expression of endogenous PC1/3). PC1/3 proteins containing the previously described S690T/Q665E (rs6234/rs6235) pair, as well as the individual S690T and Q665E SNPs, did not exhibit significantly altered expression and secretion patterns as compared to wild-type PC1/3. The N221D (rs6232) substitution resulted in reduced secretion and cleaved forms of PC1/3 in the medium (**Figure 3**). The secretion profile of the R80Q (rs1799904) substitution differed from wild-type PC1/3, in that the 74 and 66 kDa lower molecular weight forms of PC1/3 were absent from the medium (in HEK cell experiments) or reduced (in Neuro-2a cell experiments), although the total level of secreted PC1/3 was not reduced.

**Figure 3:** Western blotting of wild-type and variant PC1/3 proteins expressed in HEK cells. HEK cells were transiently transfected with empty pcDNA3 (E); pcDNA3 encoding either wild-type PC1/3; or PC1/3 proteins bearing the mutations under study. Western blots of cell lysates and media from transfected HEK cells were probed with amino-terminally directed PC1/3 primary antiserum for detection of recombinant proteins. The data shown represent 1 of 3 independent experiments performed in triplicate. Total secreted immunoreactive band intensity values, obtained through densitometry analysis and used to calculate specific activity for each variant, are represented above the Western blot and shown as the mean ± S.D.

### Catalytic activity of PC1/3 variants

To determine the impact of these variations on PC1/3 catalytic activity, conditioned medium of HEK cells transfected with either empty vector, variant PC1/3s, or wild-type PC1/3 was subjected to a fluorogenic assay. Maximum rates of fluorogenic substrate cleavage were normalized using the band intensities of secreted PC1/3s in order to determine the specific activity of each variant relative to wild-type PC1/3. The S690T/Q665E (rs6234/rs6235) and S690T (rs6234) amino acid substitutions did not significantly alter specific activity (95% confidence level; p>0.13). The Q665E substitution alone resulted in a small but significant 27% decrease in specific activity as compared to wild-type (p = 0.05). The N221D (rs6232) substitution decreased specific activity by 36% (p = 0.02), and the R80Q variation resulted in a 38% decrease (p = 0.02) (**Figure 4**). When expressed in Neuro-2a cells, the R80Q (rs1799904) variant resulted in a 42–48% decrease (p<0.0001) in activity as compared to wild-type PC1/3 (**Figure 5**).

**Figure 4:** Specific activities of wild-type and variant PC1/3 proteins, expressed in HEK cells. Enzymatic activities of secreted recombinant PC1/3 proteins in conditioned medium of transfected HEK cells were compared by measuring maximum cleavage rates using the fluorogenic substrate pyr-ERTKR-amc during a 1 h kinetic assay. Three replicates per transfection condition were assayed in triplicate, and maximum rates were divided by band intensity of immunoreactive protein in the spent medium of the same wells from which activity data were derived. Specific activity values are shown as the mean ± S.D (n = 3). Data represent one of 3 independent experiments performed in triplicate.

**Figure 5:** Western blotting of wild-type and novel R80Q (rs1799904) variant PC1/3s, expressed in Neuro-2A cells. **Panel A:** Neuro-2a cells were transiently transfected with equal amounts of empty pcDNA3 (E), or pcDNA3 encoding wild-type PC1/3 or the novel variant R80Q (rs1799904) PC1/3. Western blots of media were probed using amino-terminally directed PC1/3 primary antiserum. The data shown represent one of 3 independent experiments performed in triplicate. **Panel B: Specific activities of wild-type PC1/3 and the R80Q PC1/3 variant.** Enzymatic activities of secreted recombinant PC1/3 proteins in conditioned medium were compared by measuring maximum cleavage rates using the fluorogenic substrate pyr-ERTKR-amc during a 1 h kinetic assay. Three replicates per transfection condition were assayed in triplicate, and maximum rates were divided by band intensity of immunoreactive protein in the spent medium of the same wells from which the activity data were derived. Specific activity values are shown as the mean ± S.D. Data represent one of 3 independent experiments, each performed in triplicate.

## Discussion

In studies of European populations, *PCSK1* represents the third most important gene contributing to extreme obesity [40]. Functional studies of certain SNPs associated with obesity that impose modest or no significant effects on PC1/3 function *in vitro* have supported the idea that even slight variations in PC1/3 activity can predispose an individual to higher risk of obesity [20]. Individuals who are compound heterozygotes or are homozygous for rare severe deleterious mutations in *PCSK1* suffer from multi-dimensional disease states, including small intestinal dysfunction, hyperphagia and obesity [15], [16], [17]. Even heterozygous mutations which result in functional enzymatic changes have been linked to obesity, despite the presence of a normal allele [40]. The mechanism by which modest deficiencies in PC1/3 activity can lead to such profound phenotypes when present on a single allele remains unknown. A closer look into the complex biochemistry of commonly found variations of this enzyme may provide answers to these questions. In this work, we have analyzed public databases for other less common and rare deleterious variants and identified the variant R80Q (rs1799904), and have compared the effects of this variant to those of known polymorphisms.

Consistent with previous studies [19], [20], we found that the amino acid substitutions S690T/Q665E (rs6234/rs6235) did not significantly alter the specific activity or biosynthesis and secretion of PC1/3 in HEK cells. The Q665E substitution alone did result in a slight decrease in specific activity as compared to wild-type enzyme, and may represent the more detrimental of the two mutations (S690T/Q665E), which were previously identified as a paired SNP associated with a higher risk of developing obesity and diabetes [19], [20], [21]. In our hands, the N221D (rs6232) substitution decreased specific activity by a somewhat greater extent than previously reported, possibly due to differences in enzyme assay methods [20].

However, of all of the variants we analyzed in HEK cells, the novel R80Q (rs1799904) variant exhibited the most detrimental effects on PC1/3 maturation and specific activity. This variant yielded an 87 kDa product in the conditioned medium that did not undergo further carboxy-terminal processing to the more active 74 and 66 kDa forms, resulting in an enzyme with significantly lower specific activity, similar to the more common obesity risk N221D (rs6232) variant. This novel R80Q variant exhibited an even more pronounced decrease in specific activity when expressed in a cell line containing a regulated secretory pathway (Neuro-2a), where wild-type PC1/3 is likely able to achieve greater specific activity through more complete maturation to its lower molecular weight forms within regulated secretory vesicles. The lower molecular weight forms of PC1/3 exhibit a different substrate specificity than full-length 87 kDa PC1/3 [41]; this could be an important mechanism for SNPs to exert functional effects. Another possible functional consequence of altering the profile of active species is a change in enzyme stability, since carboxy-terminally truncated species are known to be more labile than the 87 kDa form (reviewed in [2]). Since the C-terminal region of PC1/3 has been implicated in targeting of this enzyme to secretory granules [42], [43], altered C-terminal processing may also result in changes in enzyme distribution. Further studies using immunocytochemistry in transfected Neuro- 2A cells will shed additional light on this question.

The proPC1/3 maturation process begins with the autocatalytic intramolecular cleavage of the pro-domain in the ER at the primary cleavage site, RSKR^107–110^ [44], [45]. This cleavage yields an 87 kDa form of PC1/3 that, by analogy with the related enzyme furin [46] likely remains associated with its own prodomain through non-covalent interactions until its arrival at the trans-Golgi network. Although this has not yet been strictly demonstrated for PC1/3, the PC1/3 prodomain most likely assists in the folding of the catalytic domain and in enzyme inhibition during secretory pathway transport [47], [48], [49], [50], [51], [52]. If prodomain processing of PC1/3 occurs similarly to that of furin, trans-Golgi network protonation of a histidine in the vicinity of the secondary cleavage site (RRSRR^77–81^) then results in secondary site cleavage at R^81^, followed by dissociation of prodomain fragments from PC1/3 [53], [54]. The inhibitory role of the prodomain is of particular interest to this study when we consider the location of the R80Q (rs1799904) substitution within the secondary cleavage site of the prodomain (**Figure 1**). Independent studies have shown that alteration of mouse proPC1/3 prodomain residues either within or surrounding cleavage motifs can affect propeptide processing; the *in vitro* proteolytic conversion of an R80A mutant propeptide (the same residue as the R80Q variant studied here) by wild-type enzyme was impaired compared to wild-type propeptide [44]. Given this finding, our lack of identification of propeptide-bearing R80Q PC1/3 is puzzling. We have previously found that a portion of newly synthesized proPC1/3 is subjected to endoplasmic reticulum- associated degradation [52]; this might represent the fate of this molecular species. Collectively, these data support the idea that residues within the secondary cleavage site, including the novel variant studied here, contribute to the proper processing of proPC1/3.

The novel R80Q (rs1799904) variant (MAF = 0.87%) is about one-third as common as the N221D (rs6232) SNP (MAF = 3.3%). Although less common, the R80Q variant should be subjected to further analysis to evaluate its influence on insulin sensitivity, proinsulin conversion and the risk of developing obesity, similarly to the effect of the N221D (rs6232) SNP [20], [22]. We note that 119 individuals in the public datasets have other, less common and rare variants of *PCSK1*, most of which are predicted to have some detrimental effect on protein function. This mutational burden on the population is not trivial and may also play a role in susceptibility to obesity or other disorders. The importance of rare variants in common disorders is not clear at present, but advances in massively parallel sequencing and computational analysis may soon shed additional light on this question.

In conclusion, we show that the novel *PCSK1* variant R80Q (rs1799904) exhibits deleterious effects on PC1/3 maturation. This PC1/3 variant exhibits decreased catalytic activity as compared to wild-type PC1/3 and to previously described obesity risk SNPs; therefore, it may contribute to a higher risk of metabolic disease in the general population. Our results suggest that further study of less common and rare variations in *PCSK1* from both biochemical and genetic standpoints will be useful in elucidating the mechanisms by which variant PC1/3s contribute to metabolic diseases such as obesity and diabetes.
